The article "Application of Color Doppler Ultrasound in Microscopic Imaging Diagnosis of Adenomyosis" was retracted in 2023. Reasons: unreliable results or conclusions; lack of ethics approval or compliance; concerns about the data; concerns about the peer review.

# Application of Color Doppler Ultrasound in Microscopic Imaging Diagnosis of Adenomyosis

**DOI:** 10.1155/2022/2366871

**Published:** 2022-05-31

**Authors:** Jianchang Zhu, Shuang Liu, Dandan Gao

**Affiliations:** Ultrasonic Center, Huaibei Maternal and Child Health Hospital, Huaibei Anhui 235000, China

## Abstract

In order to explore the value of color Doppler ultrasonography (TVCDS) in the diagnosis and differential diagnosis of adenomyosis. A total of 150 patients with adenomyosis admitted to a hospital from January 2020 to December 2021 were selected, taking transvaginal three-dimensional color Doppler ultrasound and abdominal ultrasound for examination, all results were compared with patient pathology or surgical results, in order to compare the accuracy of the two inspection methods. The positive predictive value of three-dimensional color Doppler ultrasonography was higher than that of abdominal ultrasonography, and the difference was statistically significant (*P* < 0.05). The coincidence rate, sensitivity, and specificity of three-dimensional color Doppler ultrasonography were higher than those of abdominal ultrasonography, while the misdiagnosis rate was lower than that of abdominal ultrasonography, and the differences were statistically significant (all *P* < 0.05). The imaging features of vaginal three-dimensional color Doppler ultrasound in patients with adenomyosis are mainly enlarged uterus, slightly stronger echoes in the myometrium with enhanced echogenic spots, and short or short branch blood flow signals in the lesions. After statistical analysis, there was a significant difference in the blood flow changes between benign and malignant endometrial echoes and abnormal echoes in the uterine cavity, *P* < 0.05. Normal endometrium and benign intrauterine lesions mainly showed no blood flow signal, while malignant lesions in the uterine cavity mostly showed changes in blood flow signal. Compared with abdominal examination, transvaginal color Doppler ultrasonography has obvious advantages in the diagnosis of adenomyosis. According to the characteristics of ultrasound images, blood flow distribution, frequency spectrum, etc., it can provide a more accurate basis for clinical timely, provide the identification points of uterine fibroids, and provide help for clinicians to choose a treatment plan.

## 1. Introduction

Uterine fibroids refer to a solid mass formed by the proliferation of smooth muscle cells, containing a small amount of fibrous connective tissue inside, with clear and smooth borders. In addition, there is a pseudocapsule composed of muscle fiber bundles and loose connective tissue. Adenomyosis is a common gynecological disease clinically, and it mostly occurred in multiparous women over 40 years old in the past, but in recent years, there is a tendency to be younger. The main cause is the invasion of endometrial glands and stroma into the myometrium, resulting in localized or diffuse lesions. Studies have shown that the disease is related to artificial abortion, cesarean section, and other surgeries [1]. There are many treatment methods for this disease, and it is necessary to choose an appropriate treatment method after comprehensive consideration of the patient's age, course of disease, reproductive requirements, and clinical symptoms. Therefore, accurate diagnosis of the disease is of great significance for physicians to choose scientific treatment methods. Clinically, histological examination and imaging examination can be used for the diagnosis of adenomyosis, histological examination is the most accurate method, imaging examination is the most effective method for preoperative diagnosis, and the process is shown in Figure 1. Clinically, the manifestations of patients with adenomyosis are quite different, a few patients do not have significant clinical features, and most patients have dysmenorrhea, therefore, it is difficult for physicians to make a diagnosis based on clinical symptoms alone [2]. Most patients with adenomyosis are found to have the disease during the process of receiving imaging tests for other diseases, or during a health check-up, for patients with adenomyosis, in the process of diagnosing adenomyosis using magnetic resonance imaging, due to its relatively high price, it has certain limitations. The three-dimensional color Doppler ultrasound has the characteristics of simplicity, convenience, and relatively low price and has gradually been widely used in clinical practice. The author mainly analyzes the clinical diagnostic value of color Doppler ultrasound for adenomyosis, aiming to provide scientific basis for the clinical examination of such diseases and provide reference value for clinical work [3].

The article "Application of Color Doppler Ultrasound in Microscopic Imaging Diagnosis of Adenomyosis" was retracted in 2023. Reasons: unreliable results or conclusions; lack of ethics approval or compliance; concerns about the data; concerns about the peer review.

## 2. Literature Review

Xu et al. indicated that adenomyosis is a relatively common gynecological disease in clinical practice, mostly in middle-aged multiparous women, and with the development of society in recent years, people's living environment is becoming more and more polluted, and work pressure is also increasing, which also leads to a younger trend of adenomyosis [4]. Mascaretti et al. stated that the etiology of adenomyosis has not yet been identified, and the consensus on the disease is that endometrial basal layer cells proliferate and invade the myometrium, accompanied by compensatory myometrial cells and hypertrophic hyperplasia [5]. Wei et al. believe that adenomyosis is related to genetics, uterine injury (cut and curettage and cesarean section), hyperestrogenemia, and other factors [6]. Cevoli et al. indicated that the clinical symptoms of adenomyosis are mainly menstrual disorders, dysmenorrhea, etc., and some patients have no obvious clinical symptoms [7]. SAFWAT and others believe that the diagnosis of adenomyosis currently mainly relies on two methods: histopathology and imaging, histopathology is the most accurate method, but its diagnosis is complex and invasive [8]. KHODAIR et al. indicated that imaging is the best preoperative diagnostic method for the disease, and transvaginal ultrasound has a high diagnostic accuracy. Magnetic resonance imaging is also a commonly used diagnostic method, which can more objectively diagnose the location and extent of lesions [9]. Shen et al. stated that the application value of ultrasonography in the diagnosis of obstetrics and gynecology diseases has been witnessed by history, and with the development of medicine and the continuous improvement of medical technology, new ultrasonography technology is widely used in various clinical disciplines. Doctors have brought convenience and speed to the diagnosis and identification of related diseases [10]. Zhi et al. stated that gynecological ultrasonography started from B-mode ultrasound, which could only be operated from the abdomen and developed to transvaginal ultrasound. The resolution of vaginal ultrasound is higher, and with the advent of color Doppler ultrasound, not only the shape of the lesions can be dynamically observed but also the blood flow in the lesions can be observed [11]. Aborizk et al. stated that in today's wide application of ultrasound examination technology and various gynecological diseases, it is essential for gynecologists to master ultrasound skills, not only the use of the final ultrasound diagnosis alone but also the characteristics of the respective ultrasound images of different uterine diseases should be able to be distinguished, which is very important for more accurate diagnosis of gynecological clinical diseases [12]. Le and others believe that in the diagnosis of gynecological diseases, ultrasound is often used as the first choice for diagnosing diseases, it can not only diagnose diseases but also a common screening method for women's health check-up, and organ diseases have high diagnostic value [13].

## 3. Methods

### 3.1. Research Overview

Color Doppler ultrasound, also known as color Doppler ultrasound, is a medical device that is suitable for ultrasound examination of various parts of the body, especially for the examination and diagnosis of the heart, limb blood vessels, and superficial organs, as well as the abdomen, obstetrics, and gynecology. Doppler ultrasound can be divided into five types: pulsed Doppler, continuous Doppler, high pulse repetition frequency Doppler, multipoint gated Doppler, and color Doppler flow imaging, among them, pulsed Doppler is the most widely used [14]. It is based on the Doppler principle and a series of electronic techniques in the case of two-dimensional echocardiography positioning, real-time display of a spectrogram of a certain volume (SV) blood flow at a certain point in the heart or great vessels. It is an atraumatic technique for detecting intracardiac shunts and regurgitation. Continuous Doppler can continuously emit pulses, so it has the ability to measure high-speed blood flow, which has obvious advantages for quantitative analysis of stenosis, regurgitation, and shunt lesions in the cardiovascular system. Its working principle is based on the introduction of color Doppler technology on the basis of high-definition black and white B ultrasound. Color Doppler ultrasound blood flow images can be formed, which not only has the advantages of two-dimensional ultrasound structural images but also provides rich information on hemodynamics. It is clinically known as “non-invasive angiography” [15]. Color Doppler blood flow imaging technology is to display blood flow signals in color, and the pseudocolor coding is composed of three basic colors of red, blue, and green. Set red to represent blood flow towards the probe and blue to represent blood flow away from the probe. Blood flow velocity is related to color luminance, with high velocity, strong color luminance, and low velocity, weak color luminance [16]. For example, when the blood flow velocity towards the probe is low, the signal is dark red, and when the blood flow velocity away from the probe is low, the signal is dark blue, the brightness of the color signal is very weak, that is, the color is very dark, and it is difficult to distinguish from the fluorescent screen. At this time, a color intensifier was added to improve the brightness of color signals in low-velocity blood flow. In order to express the speed of blood flow accurately and quickly, sometimes, three colors are used to express the speed of blood flow, the blood flow towards the probe is represented by a signal ranging from dark red to bright red, if the blood flow is faster, it will change from red to yellow, then yellow to green, and the coexistence of the three colors indicates different flow rates. Faster flow rates of blood flow away from the probe are indicated in cyan and green. On the ultrasound instrument, the color map is set to two types: one for noncardiovascular blood flow detection has only two colors of red, yellow, blue, and cyan. The other for cardiovascular blood flow detection has two to three colors in each direction. AM patients (adenomyosis patients) complete transvaginal three-dimensional color Doppler ultrasound examination before surgery, according to the imaging manifestations, the surgeon can preliminarily judge the location, size, and invasion depth of AM lesions before surgery, so as to formulate individualized surgical plan. This study shows that preoperative transvaginal three-dimensional color Doppler ultrasonography has high accuracy in diagnosing localized and diffuse AM and has a high reference value in the differential diagnosis of AM and uterine fibroids. Laparoscopic hysterectomy is used in patients with limited AM, and the recent clinical effect is definite, which can effectively relieve clinical symptoms, and is worthy of clinical application and promotion. For patients with diffuse AM, the clinical indications for laparoscopic hysterectomy wedge resection are relatively strict, mainly due to the patient's age, urgent fertility requirements, CA125 determination, etc., it is worth trying clinically, but the long-term effect needs to be further observed [17]. Research shows, other treatments, such as high-intensity focused ultrasound therapy, can also be used as a treatment option to eliminate uterine disorders and alleviate the disease process. In conclusion, transvaginal three-dimensional color Doppler ultrasound has the advantages of noninvasive, clear, measurable, etc., and it can provide specific parameter basis for the accurate diagnosis of AM types and then provide important reference indicators for the optimal selection of clinical treatment plans and postoperative follow-up, which is worthy of further application and promotion.

The article "Application of Color Doppler Ultrasound in Microscopic Imaging Diagnosis of Adenomyosis" was retracted in 2023. Reasons: unreliable results or conclusions; lack of ethics approval or compliance; concerns about the data; concerns about the peer review.

### 3.2. Data Sources

A total of 150 patients who received adenomyosis treatment in a people's hospital from January 2020 to December 2021 were selected as the research objects. The age of the patients ranged from 23 to 65 years old, with an average of (43.2 ± 2.9) years old. Among them, 25 had a history of abortion, 17 had dysmenorrhea and were infertile, and 53 had normal or slightly more menstrual flow and anemia but no history of dysmenorrhea. 55 cases of secondary dysmenorrhea. Inclusion criteria: (1) all patients were confirmed to have adenomyosis by postoperative pathology; (2) the clinical data were complete; (3) informed and agreed to this study. Exclusion criteria: (1) patients with mental illness and cognitive dysfunction; (2) patients with missing clinical data; (3) withdrew from the researcher midway.

### 3.3. Research Methods

#### 3.3.1. Ultrasound Examination

All patients underwent abdominal ultrasonography first, followed by 3D color Doppler ultrasonography, specifically: (1) abdominal ultrasound: using a color ultrasound instrument (manufacturer: Toshiba APlio, model 500), probe frequency: 5.0 ~ 9.0 MHz, before the examination, instruct the patient to drink an appropriate amount of water to ensure bladder filling, take the supine position, and test the transverse, oblique and longitudinal sections of the patient's uterus, and record the test results in detail. (2) Three-dimensional color Doppler ultrasound: put the condom on the probe and routinely sterilize it, the patient is instructed to empty the bladder before the examination, and then, the probe is slowly inserted into the patient's vagina, the oblique section, longitudinal section, and transverse section of the bladder stone were taken for examination, and the size, shape, muscle echo, endometrial thickness, and double appendages of the patient's uterus were carefully observed. Corresponding hematological tests were performed on the patients to detect the changes of blood flow in the myometrium and endometrium, and the hemodynamic index of malignant lesions was compared with the conventional hemodynamic index [18]. The above test results were analyzed and evaluated by 2 experienced laboratory personnel, and the results were compared with the surgical and pathological results.

#### 3.3.2. Observation Indicator

Taking the surgical and pathological results as the gold standard for judgment, the positive predictive value, coincidence rate, sensitivity, and specificity of the two examination methods were compared, and the main calculation methods were as follows: positive predictive value = true positives/(true positives + false positives); sensitivity = true positives/(true positives + false negatives); specificity = true negatives/(false positives + true negatives); coincidence rate = (true positives + true negatives) negative)/total number of cases [19].

### 3.4. Statistical Analysis

SPSS 18.0 software was used for statistical analysis of the data, the count data was expressed as (case (%)), the *x*^2^ test was used for data comparison, the measurement data are represented by ($\bar{x}\pm s$), the *t*-test was used to compare the data, and *P* < 0.05 was considered statistically significant.

## 4. Results and Analysis

### 4.1. Comparison of Diagnostic Efficacy of Two Ultrasound Methods

Abdominal ultrasonography was consistent in 94 cases, misdiagnosed in 27 cases, and missed in 29 cases. Vaginal three-dimensional color Doppler ultrasonography was consistent in 131 cases, misdiagnosed in 11 cases, and missed diagnosis in 8 cases, as shown in Table 1, in 11 misdiagnosed patients, when performing vaginal three-dimensional color Doppler ultrasonography, it was found that there were localized echogenic lesions in the uterine wall, and the echo was hypoechoic, which was misdiagnosed as uterine fibroids. The sensitivity, specificity, accuracy, positive predictive value, and negative predictive value of vaginal three-dimensional color Doppler ultrasound were higher than those of abdominal ultrasound, as shown in Table 2.

The article "Application of Color Doppler Ultrasound in Microscopic Imaging Diagnosis of Adenomyosis" was retracted in 2023. Reasons: unreliable results or conclusions; lack of ethics approval or compliance; concerns about the data; concerns about the peer review.

Ultrasonographic images of patients with adenomyosis diagnosed by transvaginal three-dimensional color Doppler ultrasonography, with the following characteristics: (1) the uterus has different degrees of enlargement. In diffuse adenomyosis, the uterus shows spherical enlargement, and the uterus is round and blunt. (2) There is a slightly stronger echo inside the myometrium, and the echo is uneven. (3) In some patients, echo-enhanced light spots can be seen inside the myometrium, there are two types of light spots, one is the light spot with strong and thick echoes, and the other is the anechoic or low echo area in addition to the light spot echoes. (4) There is uneven thickening of the anterior or posterior wall of the uterus, and endometrial line displacement can be seen in some patients. (5) Hematological examination showed that in the lesion, short branch-like or short-stripe blood flow signals could be seen [20].

### 4.2. Negative and Positive Comparative Analysis

Pathologically confirmed, among 150 cases of cervical lesions diagnosed by ultrasound, 91 cases (60.67%) were benign cervical lesions, and 59 cases (39.33%) were cervical malignant lesions, as shown in Figure 2.

Among the 91 cases of benign cervical lesions, 15.4% (14/91) had no obvious abnormal echoes on ultrasound, 62.6% (57/91) had hypoechoic cases, and 22.0% (20/91) had hyperechoic pathology. Among the 120 cervical malignant lesions, 16.9% (10/59) had no clear abnormal echoes on ultrasound, 79.7% (47/59) were hypoechoic, and 3.4% (2/59) were hyperechoic. Comparing ultrasound diagnosis of benign cervical lesions and malignant lesions, there was a significant difference in echo types, *x*^2^ = 82.11, *P* < 0.05, as shown in Figure 3.

Among the 91 cases of benign cervical lesions, 16 cases (17.6%), 73 cases (80.2%), and 2 cases (2.2%) showed no blood flow, punctate blood flow, and abundant blood flow, respectively, among the 59 malignant cervical lesions, there were 1 (1.7%), 19 (32.2%), and 39 (66.1%) cases with no blood flow, punctate blood flow, and abundant blood flow, respectively. After chi-square statistical analysis, there were significant differences in blood flow changes between benign cervical lesions and malignant lesions diagnosed by ultrasound, *x*^2^ = 169.56, *P* < 0.05. Benign lesions are mainly characterized by punctate blood flow, followed by no blood flow, and occasionally, abundant blood flow. On the contrary, malignant lesions are mainly characterized by abundant blood flow and punctate blood flow, but there are still a certain proportion of patients with no blood flow found in the lesions, as shown in Figure 4.

The article "Application of Color Doppler Ultrasound in Microscopic Imaging Diagnosis of Adenomyosis" was retracted in 2023. Reasons: unreliable results or conclusions; lack of ethics approval or compliance; concerns about the data; concerns about the peer review.

### 4.3. Discussion

There are many kinds of reproductive tract diseases, which affect the physical and mental health of women to varying degrees, especially uterine diseases, which not only damage the female body but also seriously affect the reproductive health of women of reproductive age; it affects the reproduction of human offspring, but if detected early, it can improve disease prognosis, improve health, and improve reproductive quality. As a simple, easy-to-operate, noninvasive, and economical examination method, ultrasound is the first choice for the diagnosis and differential diagnosis of gynecological-related diseases. How to improve the accuracy of ultrasound diagnosis of gynecological diseases is the goal that ultrasound, and clinicians have been pursuing [21]. Statistically summarizes the ultrasound imaging characteristics of uterine diseases, namely, intrauterine lesions, uterine lesions, and cervical lesions, in order to improve the detection rate of diseases, it can reduce missed diagnosis and misdiagnosis, avoid unnecessary operations or operations, and at the same time, it can also detect precancerous or malignant lesions in a timely manner, provide a reference for clinical gynecologists to accurately diagnose, design appropriate treatment plans, and select appropriate treatment methods. Ultrasound is widely used in clinical diagnosis of gynecological diseases, abdominal ultrasound is greatly affected by external factors, such as obesity, flatulence, and uterine position, it is easy to miss and misdiagnose, while hysteroscopy, hysterography, and magnetic resonance imaging have a high coincidence rate for the diagnosis of uterine diseases, but due to their relatively expensive price, complicated operation, and invasive factors such as sex limit its universality in clinical applications, therefore, transvaginal ultrasonography is widely used in clinical practice because of its noninvasiveness, simple operation, relatively low price, and high diagnostic coincidence rate. Doppler ultrasound has high diagnostic value for intrauterine lesions, uterine lesions, and cervical lesions and can be used as the first choice for disease screening; however, for the high rate of missed diagnosis of cervical lesions, ultrasound should be combined with internal diagnosis or cervical screening. Ultrasonography did not differ from MRI in assessing cervical stromal or parametrial invasion. MRI is a widely accepted and reliable method for cervical cancer detection, with the development of new ultrasound technology in recent years, ultrasound examination is also gradually used for preoperative evaluation of cervical cancer. Furthermore, ultrasonography is superior to MRI in assessing residual lesions and parametrial invasion after cervical cancer biopsy. In addition, color Doppler ultrasound can also predict the efficacy of cervical radiotherapy and chemotherapy, and not only cervical benign lesions but also cervical malignant lesions. It should be reminded that gynecological sonographers pay attention to the changes in the imaging characteristics of some cervical parts, especially the blood flow changes, which may improve the detection rate and reduce the missed diagnosis rate.

The article "Application of Color Doppler Ultrasound in Microscopic Imaging Diagnosis of Adenomyosis" was retracted in 2023. Reasons: unreliable results or conclusions; lack of ethics approval or compliance; concerns about the data; concerns about the peer review.

Transvaginal three-dimensional color Doppler ultrasound has the advantages of high resolution, noninvasiveness, sensitivity, and reproducibility, and the early diagnosis coincidence rate in AM is higher than that of abdominal color ultrasound. Transvaginal three-dimensional color Doppler ultrasound avoids factors such as excessive abdominal fat layer, uterine position, and severe pelvic gas and can accurately measure the shape, volume, muscle echo, local blood vessel distribution, and blood flow of the uterus. AM and uterine fibroids coexist in patients with localized AM (also known as adenomyoma). Ultrasound imaging features of uterine fibroids: there is a pseudocapsule around the lesion, the border of the fibroids is clear, and there may be annular blood flow signals on the pseudocapsule. Some larger uterine fibroids are prone to imaging changes of degeneration or calcification [22]. Both uterine fibroids and AM patients have clinical manifestations such as increased menstrual volume and dysmenorrhea, which are prone to misdiagnosis and missed diagnosis. However, the principles of diagnosis and treatment are different, and a clear diagnosis is required before surgery to provide basis and technical support for rational clinical diagnosis and treatment.

## 5. Conclusion

Doppler ultrasonography has high diagnostic value for intrauterine lesions, uterine lesions, and cervical lesions, and it can be used as the first choice for disease census, but ultrasound has a high rate of missed diagnosis of cervical lesions, so it should be combined with internal diagnosis or cervical screening. The results of this study show that, patients diagnosed by abdominal ultrasonography and by vaginal 3D color Doppler ultrasonography, the accuracy was significantly different, the diagnostic accuracy of abdominal ultrasound was 62.67%, and the diagnostic accuracy of vaginal three-dimensional color Doppler ultrasound was 87.33%. Sometimes due to the limited distribution of ectopic endometrium, it shows a clearer boundary with the muscle wall, but there is no dark halo around it. The blood flow in adenomyosis lesions is sparse, with a few dot-shaped short rod-shaped blood flow signals, and there is no annular or semicircular blood flow around the localized lesions, spectral Doppler detected low-speed high-resistance blood flow spectrum RI > 0.7. The main characteristics of vaginal color ultrasound imaging are the uterus is enlarged to varying degrees. There is a strong echo inside the myometrium. The enhanced echo spot can be seen inside the myometrium. Hematology showed that short strips or short dendritic blood flow signals were seen in the lesions. In summary, vaginal three-dimensional color Doppler ultrasound has a high clinical diagnostic value for adenomyosis, adenomyosis can be more accurately diagnosed, and its accuracy is significantly higher than that of abdominal ultrasonography. And because vaginal three-dimensional color Doppler ultrasound is relatively inexpensive, simple to operate, and noninvasive, it is more easily tolerated by patients. The authors believe that, under the premise of conditions permitting, this method is worthy of clinical promotion and application.

The article "Application of Color Doppler Ultrasound in Microscopic Imaging Diagnosis of Adenomyosis" was retracted in 2023. Reasons: unreliable results or conclusions; lack of ethics approval or compliance; concerns about the data; concerns about the peer review.

## Figures and Tables

**Figure 1:** Flow chart of Doppler ultrasound.

**Figure 2:** Lesion line chart.

**Figure 3:** Line chart of benign and malignant lesions.

**Figure 4:** Comparison of bleeding spots in lesions.

**Table 1:** Comparison of positive rates of abdominal ultrasonography and vaginal three-dimensional color Doppler ultrasonography.

Abdominal ultrasound	Gold standard		Vaginal 3D color Doppler ultrasound	Gold standard	
	Positive	Negative		Positive	Negative
Positive	52	21	Positive	81	14
Negative	36	41	Negative	7	48
Total	88	62		88	62

**Table 2:** The diagnostic efficiency ratio of abdominal ultrasonography and vaginal three-dimensional color Doppler ultrasonography.

Method	Sensitivity	Specificity	Accuracy	Positive predictive value	Negative predictive value
Abdominal ultrasound	68.42	51.07	64.39	31.57	60.00
3D color Doppler ultrasound	81.06	90.11	82.47	90.27	80.00

## Data Availability

The data used to support the findings of this study are available from the corresponding author upon request.
